The article "The Adsorption Potential of Cr from Water by ZnO Nanoparticles Synthesized by Azolla pinnata" was published in 2022. Journal: Bioinorg Chem Appl.

# The Adsorption Potential of Cr from Water by ZnO Nanoparticles Synthesized by *Azolla pinnata*

**DOI:** 10.1155/2022/6209013

**Published:** 2022-10-11

**Authors:** Ou Wenjie, Waqas Ahmed, Fu Xiuxian, Wang Lu, Li Jiannan, Yang Jie, Rana Muhammad Ammar Asghar, Mohsin Mahmood, Juha M. Alatalo, Muhammad Imtiaz, Weidong Li, Sajid Mehmood

**Affiliations:** ^1^Center for Eco-Environment Restoration Engineering of Hainan Province, School of Ecological and Environmental Sciences, Hainan University, Haikou 570228, China; ^2^Department of Biology, Faculty of Life Sciences, University of Okara, Punjab, Pakistan; ^3^Environmental Science Center, Qatar University, Doha, Qatar; ^4^Soil and Environmental Biotechnology Division, National Institute for Biotechnology and Genetic Engineering, Faisalabad, Pakistan

## Abstract

Aqueous solutions containing toxic elements (TEs) (such as hexavalent chromium (Cr (VI)) can be toxic to humans even at trace levels. Thus, removing TEs from the aqueous environment is essential for the protection of biodiversity, hydrosphere ecosystems, and humans. For plant fabrication of zinc oxide nanoparticles (PF-ZnONPs), *Azolla pinnata* plants were used, and X-ray diffraction (XRD), energy dispersive spectroscopy (EDS), SEM, and FTIR techniques were used for the identification of PF-ZnONPs and ZnONPs, which were used to remove Cr (VI) from aqueous solution. A number of adsorption parameters were studied, including pH, dose, concentration of metal ions, and contact time. The removal efficiency of PF-ZnONPs for Cr (VI) has been found to be 96% at a time (60 min), 69.02% at pH 4, and 70.43% at a dose (10 mg·L^−1^). It was found that the pseudo-second-order model best described the adsorption of Cr (VI) onto PF-ZnONPs, indicating a fast initial adsorption via diffusion. The experimental data were also highly consistent with the Langmuir isotherm model calculations.

## 1. Introduction

Toxic elements (TEs) stress is one of the significant abiotic stresses that have caused environmental pollution in recent decades, and their elevated concentration is highly toxic to plant [1, 2]. Currently, chromium (Cr) is one of the TEs whose concentration in the environment is still increasing alarmingly [3]. As the world's largest producer and consumer of sodium dichromate, China faces enormous environmental pressures [4]. Hexavalent chromium (Cr (VI)), besides being nonbiodegradable and highly soluble in aqueous solutions, also poses a health risk when improperly used [5]. Water containing more than 50 or 100 g·L^−1^ of Cr (VI) is considered a harmful [6]. Intakes of Cr (VI) ranging from 0.01 to 0.09 mg day^−1^ have been shown to damage the liver, kidneys, and lungs, and cause vomiting and ulcers [7]. Nearly 26 chromium production plants have been abandoned in China, and more than 40 chromium slag dumping sites exist [4]. This creates a gap in finding effective and economically feasible methods to treat TEs-contaminated water.

The article "The Adsorption Potential of Cr from Water by ZnO Nanoparticles Synthesized by Azolla pinnata" was published in 2022. Journal: Bioinorg Chem Appl.

A variety of methods are used to treat water solutions containing TEs (for example, chemical precipitation, ion exchange, and membrane electrolysis) [8]. TEs are currently treated using adsorption, a process by which molecules, ions, or atoms are bound to the surface of the adsorbent [9]. Nanomaterials are currently the most promising soil remediation agents [10, 11]. Its characteristics of a high specific variable area and strong stability can achieve the treatment of soil heavy metal pollution [12]. Because nanomaterials are insoluble in water, they also play an essential role in treating heavy metal pollution in the water [9].

Plant-based nanoparticle production is a revolutionary technique with numerous applications in agriculture, food industry, and medicine [13]. Recently, Mehmood et al. [14] suggest that silicon nanoparticles produced from *Equisetum arvense* can remove Cr (VI) pollution from affected environments in a green and innovative manner. Conventionally, synthesized NPs have limited clinical applications due to their toxicity [13]. There are many advantages to using plant-based nanoparticles compared to traditional physicochemical methods, and they are useful in a number of biological and medical applications [13]. Besides silver (Ag), copper (Cu), gold (Au), and many others, ZnO has shown potential for the biosynthesis of nanoparticles for clinical applications [15]. Researchers have synthesized ZnONPs using a variety of plant extracts, such as German chamomile, olive, and tomato extracts [16], Koseret leaf extracts [17], and beet, Malabar leaf, and cinnamon extracts [18]. We synthesized ZnONPs by *Azolla pinnata* (AP) plants.

As a biofertilizer, AP is an aquatic pteridophyte plant that fixes nitrogen in water and can be found in aquatic habitats [16]. It grows on the surface of the water with a high nutrient content [19]. In recent research, Cd, Cu, Cr, Fe, Pb, Mn, and Zn were successfully removed from the environment using *Azolla pinnata* fabricated through an adsorption [17]. By generating hydroxyl radicals in water, AP oxidizes toxic materials and shows effective results [20].

Green-synthesized nanoparticles have been used in the treatment of Cr for many years [11, 21, 22], but many challenges are yet to be overcome. An example of an in situ remediation that releases nanoparticles into the environment is the use of nanoparticles to remove contaminants [21]. The mobility and effective surface area of nanoparticles pose a toxicity risk when they are released into the environment [22]. The performance of nanoparticles should be maintained while minimizing potential disadvantages associated with their use for removing Cr (VI). An ecofriendly and simple method is presented here for manufacturing zinc oxide nanoparticles (ZnONPs) using *Azolla pinnata* as an adsorbent. The objectives of the current work were as follows: (1) produce ZnONPs from plant extract, (2) check the characteristics of produced ZnONPs and PF-ZnONPs, (3) check the effect of ZnONPs and PF-ZnONPs against Cr in the aqueous medium. Plant-fabricated zinc oxide nanoparticles (PF-ZnONPs) were characterized using X-ray diffraction (XRD), energy dispersive spectroscopy (EDS), SEM, and FTIR techniques, and their Cr (VI) adsorption potential was evaluated. Plant-based NPs can be used for sustainable crop production through this research.

The article "The Adsorption Potential of Cr from Water by ZnO Nanoparticles Synthesized by Azolla pinnata" was published in 2022. Journal: Bioinorg Chem Appl.

## 2. Materials and Methodologies

### 2.1. Experiment Materials, Chemicals, and Reagents

Anhydrous zinc sulfate (ZnSO_4_) was purchased from Xilong Science Co., Ltd. (China). Shanghai McLean Biochemical Technology Co., Ltd. (China) provided hydrochloric acid (HCl) and sodium hydroxide (NaOH). The potassium dichromate (K_2_Cr_2_O_7_) was supplied by Guangzhou Huada Chemical Reagent Co., Ltd. The absorbance of Cr (VI) was measured using a Shimadzu UV-160 spectrophotometer.

### 2.2. Plant Extract Preparation and Fabrication of ZnONPs

*Azolla pinnata* plants for ecofriendly fabrication of zinc oxide nanoparticles were purchased from a shop in Shenzhen, Guangdong, China (22°32′54.5″*N* 114°03′52.4″*E*). Plants were dried at room temperature for 4-5 days. The dried plants were then saved in polythene bags until further analysis. For the plant fabrication of ZnONPs, Jin et al. [23] methods with slight modification were followed. Following drying, 10 g of *Azolla pinnata* plants were weighed and rinsed with water. After being chopped into small pieces, the plants were soaked in 100 mL of ultrapure water in an Erlenmeyer flask for 10 minutes at 50°C. We collected, cooled, filtered the extract using filter paper, and stored it in a cold room. 20 mL of leaf extract was mixed with 20 mL of ZnSO_4_ (1 : 1, 1 M) solution and stirred at 70°C for 6 hours. NaOH (2 M) solution was used to adjust the pH to 12. Once ZnONPs were fabricated, their color changed from light yellow to white. The white precipitate was dried in an oven (Shanghai Yiheng-BPG-9240A, China) at 80°C for further analysis.

### 2.3. Characterization of Unfabricated and Plant-Fabricated ZnONPs

The pore size distribution and BET surface area for unmanufactured zinc oxide nanoparticles (ZnONPs) and plant-manufactured zinc oxide nanoparticles (PF-ZnONPs) was determined by Micromeritics Instrument Corporation (TriStar II 3020 Version 3.02 Serial ^#^2154). The micromorphological structures of ZnONPs and PF-ZnONPs were characterized by Gemini300 thermal field emission scanning electron microscope and Oxford X-MAX by energy spectroscopy and electron backscatter diffraction. The surface functional groups of ZnONPs and PF-ZnONPs were detected by iS10 FTIR spectrometer (400–4000 cm^−1^, resolution 4 cm^−1^, 64 scans) from Nicolli, USA. The crystallinity of ZnONPs and PF-ZnONPs was obtained using an XRD wide-angle diffractometer (D8 ADVANCE X-ray diffractometer, Bruker, Germany). Simultaneously, zeta potentials were measured using the Nano Brook Zeta PALS potential analyzer. Origin software version 9.1 was used to analyze all data collected from all techniques.

The article "The Adsorption Potential of Cr from Water by ZnO Nanoparticles Synthesized by Azolla pinnata" was published in 2022. Journal: Bioinorg Chem Appl.

### 2.4. Adsorption of Cr (VI) from Water Using ZnONPs and PF-ZnONPs

Several pH values, contact times, and Cr concentrations were studied in batch mode in Erlenmeyer flasks. Adsorption experiments are conducted on a pH range of 2 to 8, adsorbent amounts of 10 to 300 mg·L^−1^, contact times of 5 to 180 minutes, and Cr amounts of 20 to 100 mg·L^−1^. The solution was stirred for 12 hours with S10-3 thermostatic magnetic stirring to reach equilibrium. In order to prepare the solution for adsorption, NaOH/HNO_3_ was used to adjust the pH. Using a 0.45 m syringe filter, an aliquot was collected. A UV-vis spectrophotometer was used to measure absorbance at a 540 nm [24]. A percentage removal of Cr ions was calculated by evaluating the number of Cr ions adsorbed by the adsorbent.

(1) $$\begin{array}{c} E\%=\frac{\left(C_{o}-C_{e}\right)}{C_{o}}\times 100, \end{array}$$

where *E* represents the difference between adsorption and preadsorption metal concentration ratios.

By using the Langmuir (Eq. 2) and Freundlich (Eq. 3) equations [25], adsorption isotherm data were obtained and modeled as follows:

(2) $$\begin{array}{c} Q_{e}=\frac{Q_{m}K_{L}C_{e}}{1+K_{L}C_{e}}, \end{array}$$

(3) $$\begin{array}{c} Q_{e}=\text{Log}K_{F}+\frac{1}{n}\text{Log}C_{e}. \end{array}$$

The adsorption capacity of pollutants is given by *Q*_*e*_ (mg·g^−1^) at a specific concentration (*C*_*e*_); *Q*_*m*_ represents the maximum adsorption capacity; *K*_*L*_ (L·mg^−1^) and *K*_*F*_ (mg·g^−1^) represent Langmuir and Freundlich isotherms, respectively; *n* corresponds to the Freundlich empirical constant for adsorption strength, which fluctuates with material heterogeneity.

In order to analyze the adsorption kinetics [26], pseudo-first-order, pseudo-second-order, and intraparticle diffusion models were used.

(4) $$\begin{array}{c} Ln\left(1-\frac{q_{t}}{q_{e}}\right)=-k_{1}\times t, \end{array}$$

(5) $$\begin{array}{c} \frac{t}{q_{t}}=\frac{1}{k_{2}q_{e}^{2}}+\frac{t}{q_{e}}. \end{array}$$

*k*1 and *k*2 are the kinetic constants.

The article "The Adsorption Potential of Cr from Water by ZnO Nanoparticles Synthesized by Azolla pinnata" was published in 2022. Journal: Bioinorg Chem Appl.

### 2.5. Statistical Analysis

The adsorption investigation of Cr on ZnONPs and PF-ZnONPs was performed in triplicates. To determine the variables, the experimentally obtained % removal of chromium was analyzed using the analysis of variance (ANOVA). All experimental data were the means of three replicates. Diagrams, adsorption isotherms, and adsorption kinetic models were constructed using mean values with standard deviation. Throughout these studies, *P* < 5% was used as the level of significance.

## 3. Results and Discussion

### 3.1. Characterization of Plant-Fabricated ZnO NPs

An adsorption-desorption isotherm for N2 is shown in Figure 1, and the inset shows the pore size distribution for zinc oxide nanoparticles (ZnONPs) and plant-fabricated zinc oxide nanoparticles (PF-ZnONPs). Mesopores were found to exist in PF-ZnONPs based on the type-IV isotherm and H3 hysteresis loop [27]. Unlike the adsorption curve, the desorption curve shows a clear hysteresis loop indicating a strong interaction between the sorbent and adsorbate [28]. A BET analysis determined the average pore diameter (4 V/A) and particle size (411.70 nm) of PF-ZnONPs; their larger surface area might help bind heavy metals [29, 30]. The surface area (BET) of PF-ZnONPs was 18.99 m^2^·g^−1^. The diameter at P/Po was less than 130.99 nm and the total pore volume was 0.038 cm^3^·g^−1^. It appears that PF-ZnONPs can be a potential adsorbent for water pollution [31].

Figure 2 shows the microstructures and morphology of ZnONPs and PF-ZnONPs. SEM micrographs appear to have uniform sizes and multifaceted structures. XRD detected hexagonal structures that match this pattern. Further analysis of the structures was carried out using TEM due to the limitations of this method and agglomeration. The elemental mapping images of Zn, O, and C for ZnONPs and PF-ZnONPs are illustrated in Figure 3. EDS calculated the weight proportion of elements as 33%, 36%, and 31% for C, O, and Zn, respectively, for ZnONPs, and 52%, 29%, and 19% of C, O, and Zn for PF-ZnONPs (Figure 2). A concentration of Zn is confirmed by the elemental distribution. Water pollutants can be adsorbents with increased adsorption capacity when oxygen and carbon are present [25, 29]. TEM took images of ZnONPs, and PF-ZnONPs showed a clear adsorbent shape, size, and microstructure (Figure 4). Furthermore, the average pore diameter of the multilayered porous structure for BJH adsorption was 15.01 nm. PF-ZnONPs are capable of being adopted in real environments without compromising the adsorption capacity [31]. Figure 4 shows TEM images that confirm PF-ZnONPs have hexagonal symmetry as determined by XRD. As calculated by XRD, PF-ZnONPs have an average particle size of 20 nm. The interatomic crystallographic planes are clearly visible at a resolution of near 10 nm. A plane (101) and a plane (102) are separated by 2.42 and 1.89 A, respectively.

The article "The Adsorption Potential of Cr from Water by ZnO Nanoparticles Synthesized by Azolla pinnata" was published in 2022. Journal: Bioinorg Chem Appl.

The XRD pattern of ZnONPs and PF-ZnONPs is presented in Figures 5(a)-5(b). XRD peaks examined the crystalline mineralogy of AP, ZnONPs, and PF-ZnONPs. It was determined that (100), (002), (101), (102), (110), (103), (200), (112), (201), and (004) were polycrystalline wurtzite-structured ZnONPs and PF-ZnONPs whose peaks were measured at 31.67°, 34.31°, 36.14°, 47.40°, 56.52°, 62.73°, 66.28°, 67.91°, 69.03°, and 72.48° [26]. Crystallization of AP, ZnONPs, and PF-ZnONPs is evidenced by sharp peaks in the XRD graph [27, 32, 33]. Furthermore, FTIR analysis of ZnONPs and PF-ZnONP surfaces was conducted (Figures 6(a)-6)(b). The ZnONPs spectrum showed peaks around 1636.17, 2924.49, and 3447.75 cm^−1,^ which corresponds to C=C alkene, -C-H stretch, and carboxylic acid OH stretch, respectively [34]. While for PF-ZnONPs spectrum showed peaks around 916.66, 1509.06, 1632.86, and 3442.61, which corresponds to C-O-C, C=C aromatic, C=C alkene, and N-H stretch, respectively, [34]. There were a few CO_2_ peaks in the remaining spectrum.

In addition, the surface charges of ZnONPs and PF-ZnONPs were examined by the Zeta potential (Figure 7(a)-7(b)). According to the results, AP's surface charge was −32.9 mV, ZnONP's surface charge was −33 mV, and PF-ZnONP's surface charge was −50 mV [31, 35, 36], which shows more stability of PF-ZnONPs then other adsorbents [37]. In PF-ZnONPs, negative charge is associated with Si-OH groups [31] as SiO− species in the water deprotonate the Si-OH groups, resulting in GS-SiNPs with negative surface charges [38].

### 3.2. pH Effects

Contaminants adsorb strongly on surfaces of adsorbents based on the solution pH [39, 40]. This experiment investigated whether the pH of the solution affected the removal of Cr (VI) by changing it between 2 and 8 (Figure 8(a)). At pH 4, both PF-ZnONPs and ZnONPs effectively removed Cr (VI) at 69.02 and 69.00%, respectively (Figure 8(a)). The removal efficiency of PF-ZnONPs dropped to 67.61% and that of ZnONPs dropped to 66.92% when the pH was 7. Accordingly, PF-ZnONPs were more efficient at removing Cr under acidic conditions compared to neutral conditions, possibly due to variations in pH [41]. These results can be attributed to a number of phenomena, notably Cr (VI) reduction, and protonation and deprotonation of functional groups, depending on the pH [42]. Protonation and deprotonation of the solution as well as pH of the adsorbent were significantly correlated [43]. Under acidic conditions, PF-ZnONPs removed Cr (VI) with higher efficiency than under neutral conditions, reflecting the pH variation [41]. In a pH range of 3.0–6.0, Cr ions exist as HCrO^4−^, H_2_Cr_4_, and Cr_2_O_7_^2−^ [44]. Among Cr ions, CrO4^2−^ is the most readily reducible form at pH values of 6.0 to 12.0 [41, 45]. For further adsorption experiments, pH 4.0 was chosen. According to our study, PF-ZnONPs were able to remove Cr (VI) the least effectively at pH 2 and pH 8 (Figure 8(a)).

The article "The Adsorption Potential of Cr from Water by ZnO Nanoparticles Synthesized by Azolla pinnata" was published in 2022. Journal: Bioinorg Chem Appl.

### 3.3. Efficacy of the Adsorbent at Different Dosages

In order to remove Cr (VI), various doses of ZnONPs and PF-ZnONPs were tested (Figure 8(c)). Cr (VI) adsorption on ZnONPs and PF-ZnONPs was optimized by varying the doses of both compounds from 10 to 300 mg·L^−1^ for 60 min. It can be seen from Figure 8(c) that the removal capacity of the adsorbent decreases from 70.43% to 69.24% as PF-ZnONPs concentration increases, whereas ZnONPs decrease the adsorbent's removal capacity from 71.65% to 65.65%; this could be explained by the adsorbent containing numerous active sites [29, 31]. The surface area and adsorption potential of an adsorbent can increase as its mass increases [46].

### 3.4. Isotherm and Kinetics Analysis

During the initial 20·minutes, there was a sharp increase in Cr adsorption, but after 60 minutes, it became stable (Figure 8(b)). There is an explanation for the adsorption of Cr on ZnONPs and PF-ZnONPs that involves functional groups and active sites. In terms of PF-ZnONPs, the initial increase in adsorption rate is more likely to be caused by Cr surface complexation with functional groups than by the physical adsorption [46]. Furthermore, the adsorption behavior of Cr (VI) on ZnONPs and PF-ZnONPs was further investigated using pseudo-first- and second-order kinetic models, Figure 9.  Table 1 shows the calculated values of the relevant kinetic parameters for PF-ZnONPs. Adsorption of Cr to PF-ZnONPs and ZnONPs was well described by the pseudo-second kinetic model, suggesting valence forces and electron sharing between adsorbents and metal ions [28]. The *Q*_max_ value of ZnONPs and PF-ZnONPs was 68 and 70 mg·g^−1^, respectively.

A Langmuir and Freundlich isotherm models were fitted to the collected data to understand Cr (VI) adsorption by ZnONPs and PF-ZnONPs (Figure 10 and Table 1). The Langmuir model fit ZnONPs and PF-ZnONPs better than the Freundlich model. In the Langmuir model, *n* represents an exponential coefficient. Adsorption performance is improved by a smaller 1/*n* ratio [41]. An adsorption reaction is effective when 1/*n* ranges from 0.1 to 0.5, and it is ineffective when 1/*n* exceeds 2. This study's *n* is 0.88 for ZnONPs and 1.471 for PF-ZnONPs, indicating a favorable adsorption reaction.

The article "The Adsorption Potential of Cr from Water by ZnO Nanoparticles Synthesized by Azolla pinnata" was published in 2022. Journal: Bioinorg Chem Appl.

There are mainly two general surface complexes involved in Cr (VI) adsorption, and their configuration geometry is described by the interface configuration between sorbate and surface [47]. Adsorbate complexes can be divided into two types, inner-sphere and outer-sphere, according to whether or not they contain the hydration sphere of the adsorbate when interacting with mineral surfaces [47]. Zinc oxide nanoparticles contain hydroxyl groups on their surfaces, making them promising candidates for removing metal ions and organic contaminants [48]. In the case of Cr (VI) sorption kinetics on green nanoparticles, it was concluded that chemisorption played a critical role. Studies have suggested that Cr (VI) sorption involves a number of different interactions, such as electrostatic interactions, hydrophobic interactions, an exchange of ligands and ions, and a hydrogen bonding [14, 49, 50]. In addition, Choi et al. [51] found that the pH of the solution affected Cr (VI) adsorption and chemically altered the nanoparticle surface. Furthermore, ZnONPs and PF-ZnONPs exhibited monolayer adsorption of Cr (VI) in a homogeneous adsorption surface. It was determined that PF-ZnONPs had a maximum adsorption capacity of 60.13 mg·g^−1^, while ZnONPs had a maximum adsorption capacity of 22.89 mg·g^−1^. In terms of sorption performance, PF-ZnONPs appears to be a promising option for the removal of Cr (VI) from polluted waters. Moreover, the performance of PF-ZnONPs for removal of Cr was compared with other adsorbents in literature based on adsorption capacities and the results are presented in Table 2.

## 4. Practical Applications and Future Research Perspectives

As a result of extensive research in the green synthesis of nanoparticles over the past decade, this field has become increasingly attractive. A variety of plant extracts have already been proven to be effective for the synthesis and fabrication of materials, and their properties as stabilizing and reducing agents have been proven to be highly effective for controlled material synthesis. The purpose of this article is to provide an overview of the use of zinc oxide nanoparticles in environmental remediation for the remediation of Cr (VI). A detailed study of the synthesis mechanisms of plant-fabricated zinc oxide nanoparticles and their ability to adsorb Cr from polluted water has shown that this is a very efficient and ecofriendly way to adsorb Cr. The future of ‘green' materials and nanoparticle synthesis should extend laboratory work to an industrial scale, taking health and environmental concerns into account. However, the synthesis of ‘green' materials or nanoparticles derived from biocomponents may be applied extensively to the remediation of the environment and the pharmaceutical, food, and cosmetic industries. A significant portion of the potential of marine algae and marine plants for biosynthesis of nanoparticles remains unexplored. The synthesis of new green preparation strategies may therefore be explored.

The article "The Adsorption Potential of Cr from Water by ZnO Nanoparticles Synthesized by Azolla pinnata" was published in 2022. Journal: Bioinorg Chem Appl.

## 5. Conclusion

This investigation was conducted on zinc oxide nanoparticles and PF-ZnONPs by fabricating zinc oxide nanoparticles with *Azolla pinnata*. The parameters that affected chromium adsorption were initial Cr (VI) concentration, dose, time, and pH. When Cr concentration was increased from 20 to 100 mg·L^−1^, adsorption increased. The adsorption process followed the isotherm of Cr ion adsorption. It was found that PF-ZnONPs have a maximum adsorption capacity of 60.13 mg·g^−1^. This study shows that plant fabrication of zinc oxide nanoparticles is an ecofriendly and effective approach to adsorb Cr from polluted waters. Furthermore, these NPs also have a high adsorption capacity, making them more beneficial and cost-effective.

## Figures and Tables

**Figure 1:** Adsorption-desorption isotherms of (a) zinc oxide nanoparticles (ZnONPs) and (b) plant-fabricated zinc oxide nanoparticles (PF-ZnONPs).

**Figure 2:** SEM-EDX images of (a) zinc oxide nanoparticles (ZnONPs) and (b) plant-fabricated zinc oxide nanoparticles (PF-ZnONPs).

**Figure 3:** Elemental mappings of the homogeneous dispersion of zinc (Zn), oxygen (O), and carbon (C) elements in (a) zinc oxide nanoparticles (ZnONPs) and (b) plant-fabricated zinc oxide nanoparticles (PF-ZnONPs).

**Figure 4:** Transmission electron microscopy (TEM) images of (a) zinc oxide nanoparticles (ZnONPs) and (b) plant-fabricated zinc oxide nanoparticles (PF-ZnONPs), magnified at the accelerating voltage of 200 KV, camera length of 520 mm, and electron wavelength of 0.0251 Å.

**Figure 5:** XRD patterns of (a) zinc oxide nanoparticles (ZnONPs) and (b) plant-fabricated zinc oxide nanoparticles (PF-ZnONPs).

**Figure 6:** FTIR spectra of (a) zinc oxide nanoparticles (ZnONPs) and (b) plant-fabricated zinc oxide nanoparticles (PF-ZnONPs).

**Figure 7:** Zeta potential of (a) zinc oxide nanoparticles (ZnONPs) and (b) plant-fabricated zinc oxide nanoparticles (PF-ZnONPs).

**Figure 8:** The effect of pH on the adsorption capacity of Cr (VI) (100 mg L^−1^) at 25°C and 60 min contacting time with 100 mg L^−1^ PF-ZnONP. (b) PF-ZnONP at 25°C and 100 mg L^−1^ Cr (VI) at pH 4: effect of contact time on adsorption capacity. (c) Reduction of Cr (VI) (100 mg L^−1^) by PF-ZnONP at pH 4.0 and ambient temperature 25°C with a contact time of 60 minutes. (d) Percentage of Cr (VI) removed at different pH 4 concentrations using 100 mg L-1 of PF-ZnONP at 25°C for 60 minutes. Averages (*n* = 3) with coefficients of variation below 5%.

The article "The Adsorption Potential of Cr from Water by ZnO Nanoparticles Synthesized by Azolla pinnata" was published in 2022. Journal: Bioinorg Chem Appl.

**Figure 9:** Pseudo-first-order and pseudo-second-order equations of Cr (VI) on zinc oxide nanoparticles (ZnONPs) and plant-fabricated zinc oxide nanoparticles (PF-ZnONPs).

**Figure 10:** A plot of the Langmuir adsorption isotherm and the Freundlich adsorption isotherm of Cr (VI) on zinc oxide nanoparticles (ZnONPs) and plant-fabricated zinc oxide nanoparticles (PF-ZnONP).

**Table 1:** Experimentally determined kinetic, Langmuir, and Freundlich parameters for Cr (VI) adsorption by plant-fabricated zinc oxide nanoparticles (PF-ZnONPs).

Metric	PF-ZnONPs		
Initial Cr concentration	100 mg·L^−1^		
Contact time	60 mins		
pH	4.0		
Dosage	100 mg·L^−1^		
Langmuir isotherm	*Q*_m_ = 60.13 (mg·g^−1^)	*K*_L_ = 0.008 (L·mg^−1^)	*R* ^2^ (%) = 97.95
Freundlich isotherm	*n* = 1.471	*K*_F_ = 14.02 (mg·g^−1^)	*R* ^2^ (%) = 89.07
Pseudo-first order	*Q*_e_ (mg·g^−1^) = 53.54	K_1_ (1/min) = 0.75	*R* ^2^ (%) = 69.00
Pseudo-second order	*Q*_e_ (mg·g^−1^) = 69.95	K_2_ (g·mg^−1^·min^−1^) = 0.1	*R* ^2^ (%) = 95.00

**Table 2:** Maximum adsorption capacities of reported nano sorbent for the removal of Cr ions.

Adsorbents	Adsorption capacity (mg·g^−1^)	References
Green synthetic nano iron from tea	29.8	[52]
Eggshell-based zinc oxide nanoparticles	38.32	[53]
Orange peel nano iron	5.37	[54]
Bamboo green synthetic nano silicon	22.93	[55]
Green synthetic boehmite	59.5	[56]
Horsetail plant green synthesis of nano silicon	2.55	[15]
Fragrant pear peel nano iron	26.97	[57]
Green synthetic nano iron from eucalyptus leaves	20.5	[23]
Eggshell-based nanocrystalline chlorapatite	63.47	[58]
Biocomposite zinc oxide nanoparticles	55.56	[59]
Green synthetic nano zinc oxide from *Azolla pinnata*	60.13	This study

## Data Availability

The data used to support the findings of this study are included within the article.
